The article "Egg Incubation Mechanics of Giant Birds" was published in 2021. Journal: Biology (Basel).

# Egg Incubation Mechanics of Giant Birds

**DOI:** 10.3390/biology10080738

**Published:** 2021-08-01

**Authors:** An Yen, Hsiao-Jou Wu, Pin-Yi Chen, Hon-Tsen Yu, Jia-Yang Juang

**Affiliations:** 1 Department of Mechanical Engineering, National Taiwan University, Taipei 10617, Taiwan; yenan820812@gmail.com (A.Y.); r08b21004@ntu.edu.tw (H.-J.W.); pinyi@mit.edu (P.-Y.C.); 2 Department of Life Science, National Taiwan University, Taipei 10617, Taiwan; ayu@ntu.edu.tw; 3 Department of Mechanical Engineering, Massachusetts Institute of Technology, Cambridge, MA 02139, USA; 4 Degree Program of Genome and Systems Biology, National Taiwan University, Taipei 10617, Taiwan

**Keywords:** giant birds, contact incubation, mechanics, ratites, moa, reversed sexual size dimorphism, finite element analysis (FEA)

## Abstract

**Simple Summary:**

Extinct giant birds have been a source of imagination, and knowledge of their incubation mechanics is crucial to our understanding of the evolution of avian reproduction. Despite the extensive studies on avian eggs, our understanding of the eggshell mechanics of giant birds, particularly the extinct ones, remains incomplete—most of these prior works were based on empirical or allometric relationships with limited quantitative analysis. In the present study, with the help of advanced three-dimensional computer simulation using data from published fossil records, we obtain more comprehensive quantitative analysis to answer important questions related to contact incubation of giant birds. Specifically, how much safety margin does the reversed sexual size dimorphism (RSSD) of moas provide? What is the theoretical upper limit of body mass for contact incubation? Is the Williams’ egg, or the putative *Genyornis* oological material (PGOM), really the egg of the extinct giant bird *Genyornis newtoni*, as commonly accepted since its discovery in 1981?

**Abstract:**

Finite element analysis (FEA) was used to conduct mechanical analyses on eggshells of giant birds, and relate this to the evolution and reproductive behavior of avian species. We aim to (1) investigate mechanical characteristics of eggshell structures of various ratite species, enabling comparisons between species with or without reversed sexual size dimorphism (RSSD); (2) quantify the safety margin provided by RSSD; (3) determine whether the Williams’ egg can have been incubated by an extinct giant bird *Genyornis newtoni*; (4) determine the theoretical maximum body mass for contact incubation. We use a dimensionless number *C* to quantify relative shell stiffness with respect to the egg size, allowing for comparison across wide body masses. We find that RSSD in moas significantly increases the safety margin of contact incubation by the lighter males. However, their safety margins are still smaller than those of the moa species without RSSD. Two different strategies were adopted by giant birds—one is RSSD and thinner shells, represented by some moa species; the other is no RSSD and regular shells, represented by the giant elephant bird. Finally, we predicted that the upper limit of body mass for contact incubation was 2000 kg.

The article "Egg Incubation Mechanics of Giant Birds" was published in 2021. Journal: Biology (Basel).

## 1. Introduction

Birds have arguably been very successful in evolution [1]. In addition to the extraordinary capability of flying, they also have a special and efficient way of reproduction [2]. Most birds adopt bird-egg contact incubation and “egg turning” to maintain an adequate environment for embryonic development [2]. During such a process, eggs are subjected to the weight of the incubating bird and possible impact between eggs. Thus, paradoxically, an eggshell has to be robust enough to withstand the weight of its parent bird during incubation while also breakable for the chick to emerge; these, apparently, contradictory demands suggest an optimal design. In our previous work, we proposed a dimensionless metric, *C* number, to characterize egg stiffness with respect to egg mass. This metric facilitates the comparison of eggshell stiffness across a wide range of body mass [3]. Based on the data of 463 bird species in 36 orders across five orders of magnitude in body mass, we found that *C* number is nearly invariant for most species, including tiny hummingbirds and giant elephant birds [3]. However, that study only has limited results on giant birds, despite the fact that incubation mechanics of giant birds is crucial to our understanding of the evolution of avian reproduction.

Here, we use published data to study the incubation mechanics of ratites and an extinct giant bird *Genyornis newtoni*—a Galloansere. Ratites are large, flightless birds that are essential to understanding the early evolution of birds. The origin of the word “ratite” is the Latin word *ratis* (raft); these birds obtained their name because of their common character, a flat (raft-like) sternum without a keel to anchor wing muscles, which are necessary for flying. Ostrich, the world’s largest living bird, can be taller than a human and weigh up to 150 kg. In addition, based on fossil evidence, even larger ratite species once lived on earth. For example, the extinct elephant birds from Madagascar, the heaviest birds known to have lived, weighed up to 450 kg for the well-known *Aepyornis maximus* [4,5] and up to 650 kg for a recently recognized taxon *Vorombe titan* [6]. Both extant ratites (ostrich in Africa, rheas in South America, kiwi in New Zealand, and emu and cassowaries in Australia) and extinct ratites (moa in New Zealand and elephant bird in Madagascar) are separated from one another by oceans Figure 1. That ratites are flightless but geographically widespread has induced many discussions about their evolutionary relationships [7].

The article "Egg Incubation Mechanics of Giant Birds" was published in 2021. Journal: Biology (Basel).

According to the empirical relationship between eggshell thickness and body mass [3,8], larger birds tend to produce thicker eggshells. Therefore, the dilemma of eggshells from large-size birds may be more notable. Worthy and Holdaway [9] and Worthy et al. [10] used bone material to estimate the body mass of moa and calculated a few species reached >200 kg. Next, based on sex chromosome evidence, some moa species had reversed sexual size dimorphism (RSSD), i.e., females were larger than males [11]. For extant ratites with RSSD, e.g., emu and cassowaries, lighter males take responsibility for incubating eggs. Similarly, some researchers [8] argued that moa eggshells were not capable of withstanding the weight of the heavier sex (female), so their eggs were solely incubated by the lighter sex (male). Extreme RSSD in moa species included the strategy of compensating the mechanical discrepancy of eggshells. However, Huynen et al. [12] suggested that males of larger moa still could not perform contact incubation like extant birds. In contrast to the giant elephant bird (*Aepyornis maximus*), which had a larger size but no RSSD [6], what might be the underlying reasons for distinct mechanisms between RSSD and non-RSSD species?

Another special case related to the incubation mechanics of giant birds is the iconic Australian *Genyornis newtoni* and the issue of its associated eggshell. *Genyornis newtoni* is a Galloansere with an estimated mass of 275 kg [13]. Fossil eggshell material, known as the “Williams’ egg,” was attributed to *G. newtoni* in 1981 [14] and had been commonly accepted for many years. However, Grellet-Tinner et al. recently conducted comprehensive measurement and analysis on fossil eggshell, and concluded that this *“Genyornis*” eggshell, or the putative *Genyornis* oological material (PGOM), is unexpectedly small given the size of *G. newtoni*. They suggest that PGOM is more likely to have been laid by the giant extinct *Progura*, a genus of extinct giant megapodes. Other giant birds had also lived on earth but are now extinct. Examples include the dromornithids, gastornithids, and phorusrhacids, with some giants exceeding 500 kg [15]. Those are not included in the present study due to lack of eggshell fossils.

The objective of the present study is to use a computer simulation technique called the finite element analysis (FEA) to (1) investigate mechanical characteristics of eggshell structures of various ratite species, enabling comparisons between species with or without RSSD; (2) quantify the safety margin provided by RSSD; (3) determine whether the Williams’ egg can have been incubated by an extinct giant bird *Genyornis newtoni*; (4) determine the theoretical maximum body mass for contact incubation. Answering these questions are important to our understanding of the evolution and reproductive behavior of birds.

The article "Egg Incubation Mechanics of Giant Birds" was published in 2021. Journal: Biology (Basel).

FEA is conventionally used by engineers to design and analyze man-made structures or products, and has recently been applied to biomechanical problems in animals because of its powerful capability in predicting structure–function relationship [16]. For example, FEA has been used to infer the biting-induced stress distribution in skulls for moas (Dinornithiformes) [17], the sauropod taxa *Camarasaurus* and *Diplodocus* [18], a large carnivorous theropod dinosaur *Allosaurus fragilis* [16], the American sabercat *Smilodon fataqlis* [19], and Neanderthals (*Homo neanderthalensis*) and modern humans [20]. In our previous work, we applied three-dimensional FEA to study the eggshell mechanics of 430 avian species (36 orders, 104 families); a side-by-side comparison of eggshell stiffness of several representative species between FEA, experiments, and shell theory confirmed the accuracy of FEA [3]. This experimentally validated modelling approach was adopted here to analyze the eggshell mechanics of extinct giant birds.

## 2. Methods

Data required for our analyses, including (1) body mass, (2) egg mass, and (3) eggshell geometry (including length, width, and thickness), were obtained from the literature Table 1. Egg mass was estimated by Hoyt’s equation [21]. To increase the reliability of biological data, we gathered information from multiple sources. The eggshell geometry data of extant species was obtained from Dickison [22] and Juang et al. [3]. For extinct species, data for moa were obtained from Gill [23,24] and Worthy and Holdaway [9], whereas data for the elephant bird were from Mlíkovsky [25] and Grealy et al. [26]. Regarding body mass, we obtained not only average mass of the species but the range of both sexes, consulting three books [27,28,29], and materials from Hansford and Turvey [6], Bunce et al. [30], and Huynen et al. [12]. Note that populations of *Dinornis* (*Dinornis robustus* and *Dinornis novaezealandiae*) have markedly different size parameters for sexes [10] so our analyses are based on the correct association of egg and most relevant population data (Table 1). Population-level body mass was also used for another moa species *Emeus crassus* to ensure that its relatively low safety margin is not resulted from using unmatched species level data [23,24,31,32]. In total, data for nine extant and nine extinct avian species were collected. The data used for analyzing *G. newtoni* and PGOM were obtained from references [13,14,33,34], Table 2.

The article "Egg Incubation Mechanics of Giant Birds" was published in 2021. Journal: Biology (Basel).

### 2.1. Finite Element Analysis (FEA)

We used a finite element package ANSYS to simulate the quasi-static compression on an eggshell model along the major (long) axis, which has higher geometric stiffness [35]. Recall that the stiffness, *K* ≡ *F*/*δ*, of a load-bearing body relates to its ability to resist deformation, where *F* and *δ* are respectively the applied load and the corresponding deformation Figure 2. First, we constructed a three-dimensional eggshell model and meshed it with 4-node structural shell elements (SHELL181). The convergent test was performed to ensure that the element size was sufficiently small. We used mesh refinement around the top near where local deformation will occur due to the 0.1-N point force applied on top of the eggshell model, causing a microscopic deformation by which we obtained stiffness.

For simplicity, we assumed a perfect ellipse profile and uniform thickness. To construct an eggshell model, we used only: (1) polar diameter, (2) equatorial diameter, and (3) thickness. To save calculation time, we only created the upper half of the model and fixed the bottom ring as the boundary condition. Thereafter, the stiffness of the entire model can be obtained by dividing that of the upper-half model by two. The effect of egg content is negligible and is not included in the model [36]. The shell model is assumed linearly elastic, homogeneous and isotropic, with elastic modulus 30 GPa [3] and Poisson’s ratio 0.307 [37].

### 2.2. Dimensionless Number C, Critical Thickness, and the Factor of Safety

We used the dimensionless number defined by Juang et al. [3] as

(1) $$C\equiv \frac{A^{2}K}{BW}$$

with the length of major axis and minor axis *A* and *B*, respectively (unit: m), the weight of egg *W* in N, and stiffness *K* in N m^−1^ calculated from the FEA result. In an extreme scenario of the compression test, the eggshell is subjected to a point force equivalent to the body weight of its parent bird. By adjusting the shell thickness, the minimum thickness, referred to as the critical thickness *t_cr_*, that prevents the eggshell from buckling can be obtained (see Supplementary Figure S8 in reference [3]). We then created another eggshell model with the critical thickness, conducted the 0.1-N compression simulation again and obtained the critical dimensionless number. Note that *C* represents relative stiffness with respect to the egg size, which enables a direct comparison across a wide range of body mass. By contrast, the absolute stiffness *K* cannot be easily used for this purpose. For example, the stiffness of a massive elephant bird egg (*Aepyornis maximus*, *K* ≈ 6605 N mm^−1^) is much larger than that of a hummingbird egg (*Mellisuga minima*, *K* ≈ 11 N mm^−1^), but is it large enough to resist the incubating bird’s weight, as the elephant bird is also much heavier than the hummingbird? Interestingly, their *C* numbers are comparable (elephant bird ≈ 12,000 versus hummingbird ≈ 17,500) and similar to the average value, ~15,000, of 463 species [3]. Finally, a factor of safety, defined as the ratio of *C* to critical *C_cr_* indicates the breakability of the eggshell [3].

(2) $$F.S.\equiv \frac{C}{C_{cr}}$$

The higher the *F.S.*, the less likely the eggshell is to break (*F.S.* < 1 indicates that the parent bird cannot contact-incubate the egg without breaking it).

The article "Egg Incubation Mechanics of Giant Birds" was published in 2021. Journal: Biology (Basel).

## 3. Results and Discussion

The dimensionless number *C* can be interpreted as a measure of the stiffness of eggshell, with the geometry-induced stiffness eliminated and reflecting only contributions of shell thickness and material properties. In contrast, the critical *C* (or the further induced *F.S.*) is based on structural stability.

Scatter log-log plots for *C* number versus body mass are illustrated in Figure 3. Juang et al. [3] reported an averaged *C* of ~15,000 for 463 avian species and a slightly decreasing allometric trend of *C* with increasing body mass. Based on our results, we inferred that most ratites have a relatively lower *C* number, with ostrich (*Struthio camelus*) being an exception. Therefore, if we combined the data in Figure 3a, the slope of the blue fitting line will be slightly increased Figure 3b.

Figure 4 shows *F.S.*, *C* number, and the phylogenetic relationships of 18 ratite species, nine of which are extinct, including eight moa and one elephant bird species. Our previous study [3] shows that all of the 463 species analyzed have a *F.S.* > 2, which we adopt here as a criterion to determine the feasibility of contact incubation for extinct species. Moreover, *F.S.* in the present work was analyzed separately for the two sexes of RSSD and SSR species to investigate the feasibility of contact incubation by each sex from the mechanical point of view. Two rhea species (*Rhea americana* and *Rhea pennata*) lack sexual size dimorphism (SSD) [27], as do three moa species (*Anomalopteryx didiformis*, *Megalapteryx didinus*, and *Pachyornis elephantopus*) and elephant bird [6]. The above species were represented as green bars in the figure. Only ostrich has SSD, whereas all 11 other species are RSSD [27,38]. Costal moa (*Euryapteryx curtus*) were classified into two subspecies [39], with *Euryapteryx curtus curtus* from the North Island smaller than *Euryapteryx curtus gravis* from the South Island; they were analyzed and presented separately.

The article "Egg Incubation Mechanics of Giant Birds" was published in 2021. Journal: Biology (Basel).

An investigation of the results highlights the following observations: First, the *F.S.* values for the non-RSSD and non-SSD species (green bars) are mostly greater than two, indicating that they can contact-incubate their eggs. This is supported by the fact that two of them are extant rhea species and indeed perform contact incubation. Second, species with RSSD incubated by the lighter sex indeed provide a greater safety margin. For example, in the case of emu and the cassowaries the lighter males incubate their eggs with a safe *F.S.* > 2; the F.S. would be <2 (marginal) if the incubating sex were the heavier female. However, three moa species (*Dinornis robustus*, *Dinornis novaezealandiae*, and *Emeus crassus*) had *F.S.* < 2, even if being incubated by the lighter sex (male). Their male *F.S* was categorized as marginal, which means parent birds could perform contact incubation, but it was approaching unsafe. Furthermore, the presence of male-specific DNA on an outer eggshell supports the notion that for larger moas, their eggs were incubated by males [12]—care should be taken when interpreting this results as the shells have to be well etched before analysis to remove contaminants. In addition, based on the allometric relationship between eggshell thickness and body mass Figure 5b, the shells of the above-mentioned three moa species (*Dinornis robustus*, *Dinornis novaezealandiae*, and *Emeus crassus*) appear too thin [8]. For example, the estimated eggshell thickness of South Island giant moa (*Dinornis robustus*) ranged from 1.31 to 2.16 mm. The possibility that weathering thin the fossilized shells of those three moas was ruled out based on careful examinations of the shell cross-section of a South Island giant moa [43]; it was concluded that its shell was indeed thinner than the trend line predicted. As a result, those three moa species have *C* numbers smaller than the average of ~15,000 Figure 4c. Generally, large-size moas produced large eggs Figure 5a. If the egg was incubated by lighter males, the maternal moa could produce thinner eggshells to conserve energy. By contrast, extinct taxa with no RSSD, e.g., the elephant bird, had shell thickness 3.7 mm and *C* number ~12,000 that lie on the trend lines Figure 5b; these species had to produce stiffer eggs to withstand the weight of both parents, as compared to the RSSD moas. The elephant bird produced the largest egg (303 by 224 mm) with the thickest shell known, even larger than those of non-avian dinosaurs. Note that although ostriches exhibit SSD, both male and female birds contact-incubate their eggs, and the shell thickness, *C* number, and *F.S.* also lie on the trend lines. Thus, two different reproduction strategies have been adopted by giant birds—one is RSSD and thinner shells, represented by some moa species, emus and cassowaries; the other is no RSSD and shells with regular thickness, represented by the giant elephant bird and ostriches—the thickness of their shells follows the allometric trend in Figure 5b.

The article "Egg Incubation Mechanics of Giant Birds" was published in 2021. Journal: Biology (Basel).

### 3.1. Kiwi and PGOM

Kiwis were excluded from the fitting line due to their extreme reproductive characteristics. The kiwi is similar in height to a domestic chicken and weighs ~2 kg on average [28,44]. However, they lay an egg with approximately one-quarter of their body mass, whereas for most other avian species, the ratio of egg mass to body mass is <5%. Based on our calculations, their *F.S.* is around 2 to 5, even higher than some of the other ratites Figure 4b; they should have no problem contact-incubating eggs. However, since egg weight *W* is in the denominator of the *C* number definition, the kiwi’s large egg results in a much smaller *C* number, leading to an excessive deviation from the allometric trend Figure 4c.

Another special case herein is an extinct Australian avian species, *Genyornis newtoni*, which exhibits SSD with the smaller and larger sexes having an estimated mean mass of 192.8 kg (range 180–203 kg) and 238.4 kg (range 214–262 kg), respectively [33]. Grellet-Tinner et al. [13] suggested that an extinct large megapode, which belonged to the genus *Progura*, was more likely to be the parent bird of the putative *Genyornis* oological material (PGOM, to use their abbreviation), which was assigned to *Genyornis* by Williams [14], a conclusion accepted for decades. Shute et al. [34] taxonomically described/revised several large extinct megapodes from Australia. The species of *Progura* mentioned by Grellet-Tinner et al. [13] were classified as separate species called *Latagallina naracoortensis* and *Progura gallinacea*. In the calculation of *C* number and *F.S.* for PGOM, we used the two above-mentioned species and *Genyornis newtoni*, then computed with Williams’ egg [14] and the egg of Grellet-Tinner et al. [13], the so-called Spooner egg (126 by 97 mm). In addition, Grellet-Tinner et al. suggested that the size of the complete shell of Williams’ egg (155 by 125 mm), estimated based on shell curvature, may have been overestimated [33]. They considered that Williams’ egg might be the same length and width as the Spooner egg. Therefore, we additionally simulated the specimen with length and width of the Spooner egg but using the shell thickness of the Williams’ egg. Figure 3d shows the *C* numbers of various egg-bird combinations. The combination of Williams’ egg and *Genyornis newtoni* lies on the allometric trend line, whereas the combinations of the Spooner egg and the two megapodes were consistent with the trend. However, the *F.S.* values of *Genyornis newtoni* are <1, suggesting that neither the Williams’ egg nor the Spooner egg could be contact incubated by *Genyornis newtoni*. On the other hand, the *F.S.* values of the two extinct megapodes are >2 and are even higher than those of some extant counterparts Figure 6, which suggests that megapodes may have evolved a less stiff eggshell to adapt to their new environment during the Pleistocene era. Accordingly, we conclude that the Williams’ egg is unlikely associated with *Genyornis newtoni* and is likely to be the egg of extinct megapodes with a dimension similar to the Spooner egg’s. Table 3 lists eggs of extant birds that have similar size to the Spooner egg for comparison.

The article "Egg Incubation Mechanics of Giant Birds" was published in 2021. Journal: Biology (Basel).

### 3.2. Maximum Body Mass for Contact Incubation

When considering the maximum body mass of avian species, the egg is assuredly an important factor [5]. Deeming and Birchard [45] proposed that contact incubation prevents avian species from attaining great sizes. In addition, they also explained that extinct “gigantic” birds were not truly gigantic, compared to mammals and non-avian dinosaurs. Finally, they proposed a maximum mass of 500 kg.

In this study, we estimate the maximum avian body mass by considering the body mass at which the allometric line of *F.S.* becomes smaller than one—contact incubation is no longer possible. Recall that *F.S*. ≡ *C*/*C_cr_* and from Figure 3b we observe that the two solid fitting lines for *C* and *C_cr_* intersect at ~2000 kg, which may be regarded as an estimate of the theoretical upper limit of body mass for contact incubation. This estimate, of course, may vary within a certain range according to the dash lines of 95% confidence interval. Note that the critical thickness was defined by considering the failure mode of buckling instead of fracture. The former is easier to predict, whereas the latter is sensitive to micro-cracks and thus not easy to determine [3,36]. Since the buckling force is generally greater than the fracture force, i.e., an egg under compression fractures before buckling, our upper limit was assuredly high enough to be a valid estimate. It is noteworthy that 2000 kg is well above the maximum estimated mass for the largest known birds, e.g., *Vorombe titan*, ~650 kg. Such a discrepancy might be explained by the fact that our analysis only considers whether an eggshell is strong enough to sustain the weight of the incubating bird. Another key factor that constrains the maximum body size—the hatching process—is not considered in the present study. Larger eggs have thicker shells, and result in a more challenging and prolonged hatching process. For example, it can take several hours for an ostrich chick to hatch naturally. In other words, the allowable body mass (and thus the maximum egg size) for contact incubation, constrained by hatching mechanics, is likely lower than 2000 kg. As an interesting analogy, gigantic size of 2000 kg or heavier is not rare and has been achieved by extinct and extant mammals, as well as many theropod dinosaurs—close relatives of birds. One reason they can evolve such gigantic sizes, compared to birds, is that they are not constrained by mechanics of contact incubation.

The article "Egg Incubation Mechanics of Giant Birds" was published in 2021. Journal: Biology (Basel).

## 4. Conclusions

Size is a critical factor in evolution. Although extensive research on allometry related to avian reproduction has been performed, our research provides mechanical analyses on eggshells of both extant and extinct ratites and galloanseres. Based on our data, RSSD in moas significantly increases the safety margin of contact incubation if the incubation is indeed conducted solely by the lighter males. However, their safety margins are still, in general, smaller than those of the moa species without RSSD. Thus, two different reproduction strategies have been adopted by giant birds—one is RSSD and thinner shells, represented by some moa species, emus, and cassowaries; the other is no RSSD and shells with regular thickness, represented by the giant elephant bird and ostriches. In addition, our FEA shows that the Williams’ egg could not be contact incubated by *Genyornis newtoni* and is more likely associated with an extinct species of megapodes. Finally, we proposed a theoretical upper limit of body mass, ~2000 kg, for contact incubation based on numerical simulation (*F.S.* = 1). One of the most important obstacles of investigating extinct species is that materials are insufficient since fossil formation and discovery are both incidental. Regardless, our model can be used as a tool to analyze additional fossil evidence, obtained either by using DNA sequences to identify those eggshell fragments previously unidentified or by discovering new eggshell fragments accompanied by their respective adult skeleton, and thereby strengthen the allometric relationship. The mechanisms of evolution are inherently complex. In that regard, specific species might deviate from the allometric trend to some extent due to particular adaptations (e.g., kiwis, as mentioned above). However, if we assess a large range across body mass of many orders of magnitude, the interspecific allometric trend indeed provides some evolutionary insights regarding reproductive strategies of oviparous animals laying eggs protected by hard shells.

The article "Egg Incubation Mechanics of Giant Birds" was published in 2021. Journal: Biology (Basel).

## Figures and Tables

**Figure 1:** Extant distribution of living ratites and the Holocene distribution of moa and elephant birds. Each color relates the ratite groups to their area of origin. Kiwi birds, which range from 10–100 kg, are printed in gray color. Silhouettes of birds and eggs indicate a relative proportion of actual size. RSSD or SSD is implied by marking sex symbols on two different silhouettes within a species. For species without significant RSSD or SSD, there is only one silhouette. See Supplementary Materials Dataset Table S1 for details on the source of bird images.

**Figure 2:** Eggshell models in finite element package ANSYS (Mechanical APDL 15.0). (**a**) a representative mesh of the upper-half eggshell with mesh-refinement near the top. The bottom ring (equator) is fixed. (**b**) a cross-sectional view of the displacement field in the *y*-direction (upward) subjected to a point load, *F*, on top. Negative value, marked in blue, represents downward displacement. *δ* is the displacement at the load application point. This particular case demonstrates the scenario of critical thickness.

**Figure 3:** Allometries between body mass (BM) and the dimensionless number *C* (blue) and critical *C* (red) on a double logarithmic scale. Dash lines: 95% confidence interval. (**a**) two fitting lines of data from Juang et al. [3] with data points of 15 ratite species (excluding kiwi, see discussion). (**b**) new fitting lines combined with data points of 15 ratite species. (**c**) the new fitting line of *C* with three data points of kiwi. (**d**) the new fitting line of *C* with six data points of PGOM. Williams’ egg is marked as a light blue star, whereas the Spooner egg is marked as a red star. Purple hollow stars indicate our additional specimens. Points of larger body mass represent *Genyornis newtoni*, whereas smaller points represent two extinct megapodes, respectively.

**Figure 4:** Factor of safety *F.S.*, *C* number and the phylogenetic relationship of 18 ratite species. The phylogenetic tree was plotted with cladogram using ggtree [40,41] and the nearby graph was plotted by package ggplot2 [42]. (**a**) phylogeny of ratites is based on a tree of Mitchell et al. [7], and phylogeny of moa is supplemented by Bunce et al. [30]. (**b**) the pink bar indicates the case of incubation by females, whereas blue indicates incubation by males. The purple bar in some species indicates *F.S.* overlap of two sexes, whereas green indicates species with no sexual size dimorphism. (**c**) the *C* numbers for ratites were predicted by FEA simulations. See Supplementary Dataset for details on the source of bird images (Table S1).

The article "Egg Incubation Mechanics of Giant Birds" was published in 2021. Journal: Biology (Basel).

**Figure 5:** The regression line of (**a**) initial egg mass and (**b**) eggshell thickness on body mass. Data used to plot regression are from Juang et al. [3]. Green dots indicate species with no RSSD. Red dots (female) and blue dots (male) connected by dashed lines indicate species with RSSD. The numbers 1 to 18 represent different species, as denoted in Table 1.

**Figure 6:** Factor of safety *F.S.*, *C* number and the phylogenetic relationship of megapodes and *Genyornis newtoni*. (**a**) phylogenetic tree of megapodes is based on Shute et al. [34]. (**b**) *F.S.* of extinct species were calculated with Williams’ egg (red), Spooner egg (blue), and additional specimen (yellow), respectively. Extant megapodes are illustrated as black dots. (**c**) different colors of *C* number indicate identical implication of *F.S.*

**Table 1:** Absent of MBM indicates that species with no SSD or RSSD. FBM: female body mass (kg), MBM: male body mass (kg), and ESR: egg size ratio (egg mass divided by average body mass). *^a^* cassowary, *^b^* emu, *^c^* kiwi bird, *^d^* ostrich, *^e^* rhea, *^f^* elephant bird, *^g^* moa.

Species	Egg Length, *B* (mm)	Egg Width, *A* (mm)	Shell Thickness, *t* (mm)	Egg Mass, *W* (g)	Body Mass, *M* (kg)				ESR	Ref.
					FBM (Max.)	FBM (Min.)	MBM (Max.)	MBM (Min.)		
*^1^ Struthio camelus ^d^*	158	131	1.92	1600	85	63	130	80	1.79%	[3,12]
*^2^ Rhea americana ^e^*	128	86	0.9	525	40	20			1.75%	[3,28]
*^3^ Rhea pennata ^e^*	126	92	0.86	584	25	15			2.92%	[22,28]
*^4^ Dromaius novaehollandiae ^b^*	136	89	0.94	610	45	35	30	20	1.88%	[3,12]
*^5^ Casuarius casuarius ^a^*	135	92	0.97	644	50	35	30	25	1.84%	[3,12]
*^6^ Casuarius unappendiculatus ^a^*	136	90	0.97	604	64.35	52.65	40.7	33.3	1.26%	[22,27]
*^7^ Apteryx owenii ^c^*	110	70	0.4	295	1.9	1	1.3	0.9	23.17%	[22,28]
*^8^ Apteryx haastii ^c^*	123	77	0.53	400	3.3	1.5	2.6	1.2	18.59%	[22,28]
*^9^ Apteryx mantelli ^c^*	125	78	0.5	417	3.27	2.09	2.59	1.82	17.06%	[22,27]
*^1^* *^0^ Aepyornis maximus ^f^*	303	224	3.7	9120	541	334			2.08%	[6,25,26]
*^11^ Megalapteryx didinus ^g^*	160	108	1.17	1023	80	28			1.89%	[23,30]
*^12^ Dinornis novaezealandiae ^g^*	190	150	1.375	2343	160	91	69	34	2.65%	[10,23,24]
*^13^ Dinornis robustus ^g^*	240	178	1.23	4167	275	102	113	61	3.03%	[10,23,24]
*^14^ Pachyornis elephantopus ^g^*	221	150	1.79	2725	106	49			3.52%	[23,29]
*^15^ Anomalopteryx didiformis ^g^*	165	120	1.39	1302	64	26			2.89%	[23,30]
*^16^ Euryapteryx curtus curtus ^g^*	121	97	0.9	624	30	20	20	15	2.94%	[12,23]
*^17^ Euryapteryx curtus gravis ^g^*	205	158	1.5	2804	105	67	80	55	3.65%	[12,23]
*^18^ Emeus crassus ^g^*	179	134	1	1761	80	52	50	36	3.23%	[23,24,31,32]

Note: Data used in the simulation.

The article "Egg Incubation Mechanics of Giant Birds" was published in 2021. Journal: Biology (Basel).

**Table 2:** Comparison of two known eggs (with measured parameters) with possible source taxa (with estimated body mass) to generate ESR. These values were used in the FEA simulations. ESR: egg size ratio (W/M).

Egg Specimen	Species	Egg Length, *B* (mm)	Egg Breath, *A* (mm)	Shell Thickness, *t* (mm)	Egg Mass, *W* (g)	Body Mass, *M* (kg)	ESR	Ref.
Williams	*Genyornis newtoni*	155	125	1.15	1327	192	0.69%	[14,33]
	*Latagallina naracoortensis*	155	125	1.15	1327	6.1	21.75%	[13,14,34]
	*Progura gallinacea*	155	125	1.15	1327	7.7	17.23%	[13,14,34]
Spooner Egg	*Genyornis newtoni*	126	97	1.3	650	192	0.34%	[13,33]
	*Latagallina naracoortensis*	126	97	1.3	650	6.1	10.66%	[13,34]
	*Progura gallinacea*	126	97	1.3	650	7.7	8.44%	[13,34]

**Table 3:** Similar eggshell geometries with PGOM (putative *Genyornis* oological material). Data were published by Juang et al. [3]. The bold text indicates similarity to the Spooner egg <15%. (Length: 126 mm, width: 97 mm).

Species	Common Name	Egg Length, *B* (mm)	Egg Width, *A* (mm)	Shell Thickness, *t* (mm)	Egg Mass, *W* (g)	Body Mass, *M* (g)	Dimensionless Number, *C*	Factor of Safety, *F.S.*
*Diomedea Exulans*	Wandering Albatross	**129.5**	**79.7**	0.58	455.0	8190	3185	2.16
*Phoebastria Nigripes*	Black-footed Albatross	**108.2**	69.2	0.50	286.0	3195	6328	4.81
*Phoebetria Palpebrata*	Light-mantled Albatross	**104.0**	64.5	0.48	243.0	3150	5428	3.95
*Macronectes Giganteus*	Southern Giant Petrel	**104.4**	65.9	0.58	237.0	4395	10,865	5.61
*Aptenodytes Patagonicus*	King Penguin	**104.5**	75.8	0.80	306.0	11,751	13,741	4.00
*Cygnus Columbianus*	Tundra Swan	**106.9**	68.2	0.76	280.0	6750	12,655	2.41
*Pinguinus Impennis*	Great auk	**124.0**	75.8	0.74	372.0	5000	8299	7.56
*Rhea Americana*	Greater Rhea	**128.0**	**86.0**	0.90	525.0	23,000	9637	2.80
*Casuarius Casuarius*	Southern Cassowary	**135.0**	**92.1**	0.97	644.0	44,000	9108	2.12
*Dromaius Novaehollandiae*	Emu	**136.0**	**89.0**	0.94	610.0	34,200	8043	2.02
*Apteryx Australis*	Southern Brown Kiwi	**125.8**	**78.5**	0.50	434.0	2330	3924	2.79
*Macrocephalon Maleo*	Maleo	**105.6**	61.7	0.38	222.0	1564	3488	3.20
*Gymnogyps Californianus*	California Condor	**110.2**	66.7	0.92	280.0	8450	17,911	6.08

## Data Availability

The data presented in this study are available on request from the corresponding author.

## Supplementary Materials

The following are available online at https://www.mdpi.com/article/10.3390/biology10080738/s1, Table S1: copyright information about bird images.
